# Diagnostic Value of Magnetic Resonance Imaging Scan, Multislice Spiral Computed Tomography Three-Dimensional Reconstruction Combined with Plain Film X-Ray in Spinal Injuries

**DOI:** 10.1155/2022/8998231

**Published:** 2022-05-16

**Authors:** Dajiang Xin, Lei Lei

**Affiliations:** ^1^Department 3 of Trauma, Yantai Mountain Hospital, Yantai City 264000, Shandong Province, China; ^2^Department of Medical Imaging, Hohhot First Hospital, Hohhot City 010059, Inner Mongolia Autonomous Region, China

## Abstract

**Objective:**

The main objective is to explore the diagnostic value of magnetic resonance imaging (MRI) scan, multislice spiral computed tomography (MSCT) three-dimensional reconstruction combined with plain film X-ray in spiral injuries.

**Methods:**

By means of retrospective study, the data of 100 patients with spiral injury treated in our hospital from January 2020 to December 2021 were retrospectively analyzed, and all patients received MRI scan, MSCT three-dimensional reconstruction, and plain film X-ray examination, and by taking the operation results as the reference, the diagnostic results of different diagnostic modalities were analyzed, and the accordance rates (diagnostic result/surgical result × 100%) of the three diagnostic modalities and their combination were calculated, respectively.

**Results:**

Among the 100 patients, 52 cases (52%) had a fracture at the anterior column of the spine, 28 cases (28%) had a fracture at the middle column of the spine, and 20 cases (20%) had a fracture at the posterior column of spine; 24 cases (24%) had simple flexion compression fracture, 60 cases (60%) had burst fracture, 6 cases (6%) had seat belt fracture, and 10 cases (10%) had fracture dislocation. The accordance rate of combined diagnosis for fracture site was 100%, and that for fracture type was 98.0%; MRI could visualize bone marrow injuries, ligamentous injuries, soft tissue injuries, and nerve root injuries that could not be visualized on X-ray plain films, and 3D reconstruction with MSCT could clearly demonstrate the 3D relationship of spinal fracture displacement, fracture line orientation, and spinal injury.

**Conclusion:**

Plain film X-ray is the basic method for diagnosing spinal injuries, while MRI and MSCT have their unique advantages in this regard, and patients with a negative result of X-ray plain film can be examined by MRI and MSCT to observe the spinal injury comprehensively.

## 1. Introduction

Spinal injuries, which result from indirect or direct external forces, are a common type of injury in the clinic [1]. Because of the complex anatomical structure, spinal injuries can cause curvature changes, displacement of fracture fragments, ligamentous injuries, soft tissue changes around the fractured vertebral bodies, etc., and for severe cases who are complicated with spinal cord injury (SCI), their movement, reflexes, and sphincters below the injury plane will be impaired [2, 3]. With the lifestyle changes of Chinese residents, the cause of injury to the spine has gradually increased, and the situation of spinal fractures is becoming more complex, so an accurate diagnosis of the site and type of spinal injuries in patients is beneficial to orthopedic physicians to develop the corresponding treatment plan, which is of great importance to reduce the disability and mortality of patients [4]. Plain film X-ray is the conventional diagnostic modality of spine injuries, which can clarify the compression of the vertebral body at the injured part, but may easily miss the cases with less severe compression [5], especially in patients with long-standing pain after trauma, X-ray plain films often fail to show the fracture signs, and they are usually diagnosed with soft tissue contusion, delaying their treatment time [6]. The current application of magnetic resonance imaging (MRI) and computed tomography (CT) further highlights the disadvantages of X-ray plain films, and more and more physicians prefer to choose MRI and CT to diagnose the injury condition of the spine [7, 8]. MRI has a unique diagnostic advantage for SCI, because paraspinal ligaments, disc injury, and paraspinal hematoma can only be detected by MRI, whereas conventional CT can only rely on the indirect signs to judge bone marrow and soft tissue injuries, with a poor clinical detection rate. The promotion of multislice spiral computed tomography (MSCT) in recent years has led to the improvement of CT examination results, and MSCT three-dimensional reconstruction can remove other bones and soft tissues, thus clearly showing the stereo image of the spine, facilitating physicians to observe the fracture line course in a full range and at many angles, and providing a good basis for determining the surgical plan and surgical path in the clinic [9]. At present, there are no studies in academia that combine plain film X-ray, MRI, and MSCT 3D reconstruction, but they all have their own advantages in diagnosing spinal injuries, and their combination may complement each other's advantages, improving the accuracy of spine injury diagnosis. Based on this, 100 patients with spinal injury were chosen as the subjects to explore the diagnostic value of combining MRI and MSCT three-dimensional reconstruction with plain film X-ray in spinal injury.

## 2. Materials and Methods

### 2.1. General Data

The data of spinal injury patients treated in our hospital from January 2020 to December 2021 were retrospectively analyzed, and 100 patients over 18 years old with a clear history of acute spinal trauma were selected, including 68 males and 32 females, with a mean age of (49.41 ± 8.90) years and a mean course of disease of (1.95 ± 0.71) d, and in terms of the cause of injury, 15 cases were caused by high-altitude falling, 30 cases were caused by a traffic accident, 38 cases were caused by a fall on the flat ground, 12 cases were caused by damage from the heavy object, and 5 cases were caused by other factors. All 100 patients presented with varying degrees of spinal pain and limited mobility, including 15 with paralysis of the lower extremities. All patients required surgical treatment and had the good cognitive ability to go along with MRI scan, MSCT three-dimensional reconstruction, and plain film X-ray examination.

Patients with spinal injury due to other reasons [10], with contraindications of relevant imaging examinations [11], complicated with other severe organic diseases and in pregnancy or lactation were excluded from the study.

### 2.2. Moral Consideration

The study was conducted under the guidance of the World Medical Association Declaration of Helsinki [12], and the patients and their family members understood the study objective, meaning, content, and confidentiality and signed the informed consent.

### 2.3. Methods

#### 2.3.1. MRI Scan

The GE Signa Excite 1.5T superconducting MRI instrument (NMPA Registration (I) no. 20153333982) was used, patients were kept in a proper position with assistance, cervical coil and spinal surface coil were selected, and axial, sagittal, and coronal scans were determined based on the site of the spinal lesion in the patients, with the parameters of SE T_1_WI TR/TE = 400/12 ms, FSE T_2_WI TR/TE = 3200/105–120 ms, STIR TR/TE = 4000/56 ms, slice thickness of 4.0 mm, slice gap of 4.0 mm, interval of 1 mm, and 256 × 256 matrix.

#### 2.3.2. MSCT 3D Reconstruction

The Philips MSCT scanner (NMPA Certified No. (2018) 3303600) was used, the patients were in the spine position with assistance, and ROIs were selected for scan based on the positioning image, with the set slice thickness of 2.5 mm, thin-layer reconstruction slice thickness of 2.0 mm, reconstruction interval of 1.5 mm, pitch of 1.5, tube voltage of 120 KV, and tube current of 120 mA. The acquired original cross-sectional CT images were transferred to a Philips Brilliance Workspace 2.0 workstation for 3D reconstruction, including multiplanar reconstruction volume reproduction (VR), with the built-in processing software. VR images hid the tissues that were not associated with the bone through adjustment of the threshold to clearly reveal the bones.

#### 2.3.3. Plain Film X-Ray

The X-ray apparatus made by Shanghai Xin Huang Pu Medical Equipment Co., Ltd. (Shanghai Medical Products Administration Certified No. 20132301725) was used to regularly shoot the positive lateral plain film of the spinal segment at the lesion site, and the plain films of double oblique view were taken for some patients.

### 2.4. Observation Criteria

According to the three-column concept for classification [13], spinal injuries are divided into four types, that is, (1) simple flexion compression type, (2) burst type, (3) seat belt type, and (4) fracture-dislocation type.

The slides were read jointly by 2 radiologists and 1 orthopedic surgeon under double-blind conditions, and they reached a consensus conclusion through discussion. The results of the surgery were set as the standard in both groups, and the accordance of the results of imaging examinations with the standard was determined.

### 2.5. Statistical Processing

In this study, the data processing software was SPSS20.0, the picture drawing software was GraphPad Prism 7 (GraphPad Software, San Diego, USA), the items included were enumeration data and measurement data, the methods used were *X*^2^ test and *t*-test, and differences were considered statistically significant at *P* < 0.05.

## 3. Results

### 3.1. Analysis of Results of Imaging Examinations

MRI. Vertebral fractures were shown as displacement of the vertebral bone fragments towards the front, displacement of the bone scraps at the posterior border into the posterior spinal canal, increased signal within the vertebral body, low or equal signal on T_1_WI, and high signal on T_2_WI. According to the MRI findings, 48 cases had injury of anterior ligament, which revealed as thickened anterior longitudinal ligament and increased signal on T_2_WI and STIR; 24 cases had injury of posterior ligament, which revealed as thickened posterior longitudinal ligament and increased signal on T_2_WI and STIR; 63 cases had SCI, with longitudinal strip isointensity and hypointensity in the spinal cord on T_1_WI, slightly high signal on T_2_WI, high signal on STIR, heterogeneous signal, and increased volume of the spinal cord in the injured segment; and 76 cases had injury of soft tissue, with patchy hyperintensity on T_2_WI and STIR, and slightly low signal on T_1_WI.

MSCT. Vertebral fractures were shown as flattening of the vertebral body with a wedge-shaped appearance, and in 82 cases, the fracture line and displaced bone were visible. The 3D reconstruction of MSCT could not fully reflect SCI, and only partial swelling and hemorrhage within the spinal cord could be revealed. MSCT only showed anterior longitudinal ligament thickening in 10 cases and posterior longitudinal ligament thickening in 8 cases, while the ligament injury in the remaining cases was failed to show directly.

*X-Ray Plain Films.* The fracture line appeared sharp in the lateral X-ray film. X-ray plain films failed to reveal injuries of the anterior ligament, posterior ligament, and spinal cord.

In short, MRI can reveal bone marrow injury, ligament injury, soft tissue injury, and nerve root injury that cannot be visualized on X-ray plain films, and MSCT 3D reconstruction can clearly demonstrate the 3D relationship of spinal fracture displacement, fracture line course, and spinal injury (see Table 1 for the analysis of the results of the three imaging examinations).

### 3.2. Comparison of Accordance Rates of Imaging Examinations

According to the three-column concept, among the 100 patients, 52 cases had fracture at the anterior column of the spine, 28 cases had fracture at the middle column of the spine, and 20 cases had fracture at the posterior column of the spine; 24 cases had simple flexion compression fracture, 60 cases had burst fracture, 6 cases had seat belt fracture, and 10 cases had fracture dislocation. The accordance rate of combined diagnosis for fracture site was 100%, and that for fracture type was 98.0% (see Table 2).

## 4. Discussion

Spinal injuries occupy an important position in systemic osteoarticular injuries, and vertebral fractures are more common in the clinic, accompanied by adnexal fractures in some patients, and their fracture rate is approximately 5.0%–6.0% of patients with systemic fractures [14]. Since the spine is a complex structure with multiple bones, in which joints and nerves are intricate, fracture patients may also suffer from complications such as SCI and nerve injury, which, in severe cases, seriously affect the physiological function of their internal organs and even make them lose the function of lower limbs and face the risk of paralysis or death [15, 16]. Accurate judgment of spinal injuries is beneficial for orthopedics to make surgical plans and improve patient outcomes, so intuitive and practical diagnostic modalities should be chosen in practice to enhance the diagnostic accuracy of spinal injuries. Plain film X-ray is the most basic diagnostic modality for spinal injuries, which can directly reflect the injured part in patients with vertebral fractures and is inexpensive, presenting a wide market value [17]. With the assistance of plain film X-ray, physicians can comprehensively analyze information such as the degree of compression and the interpedicular distance of the injured vertebral bodies of patients, so as to judge the fracture type. However, plain film X-ray is subject to the influence of spinal structure and cannot adequately detect fractures at overlapping sites, and in particular, it is difficult for plain film X-ray to distinguish whether the spinal canal is involved or not, and whether there is damage to soft tissues [18–20]. In this study, plain film X-ray failed to show the injuries of the anterior ligament, posterior ligament, and spinal cord. The utility of plain film X-ray is further limited by the complex patient condition, and there are often instances in practice in which patients are symptomatic and obtain negative X-ray results. To make up for the deficiencies of plain film X-ray, physicians usually advocate performing additional MRI or CT for patients with negative X-ray result [9]. MRI, due to its high soft-tissue resolution, can be used to accurately determine the injuries of soft tissue, ligament as well as bone marrow, and especially simple bone marrow injury and ligament injury. Scholars Shah et al. found that at the early stage of ligament injury, MRI showed low signal on T_1_WI and T_2_WI, and the signal was more uniform [21]. According to the MRI findings of the study, 48 cases had injury of anterior ligament, which revealed as thickened anterior longitudinal ligament and increased signal on T_2_WI and STIR, and 24 cases had injury of posterior ligament, which revealed as thickened posterior longitudinal ligament and increased signal on T_2_WI and STIR. Bone marrow injury, as the most serious complication of spinal injury, can manifest as spinal cord edema, hemorrhage, contusion, and its early diagnosis can only be made by MRI [22]. Spinal cord lesions on MRI generally appear as longitudinal strips, patchy equal signals, or low signals. The MRI findings in this study showed that 63 cases had SCI, with longitudinal strip isointensity and hypointensity in the spinal cord on T_1_WI, slightly high signal on T_2_WI, high signal on STIR, heterogeneous signal, and increased volume of the spinal cord in the injured segment; in addition, 76 cases had injury of soft tissue, with patchy high signal on T_2_WI and STIR, and slightly low signal on T_1_WI.

Although MSCT had a detection rate for SCI and soft tissue injury inferior to that of MRI, it has the advantage of stereological imaging to adequately exclude overlapping interference [23]. MSCT has an independent postprocessing work station and includes a variety of reorganization ways, which can obtain the 3D images of bone and joint structure with only the cross-sectional data of CT, and physicians can observe the overall situation of fracture by 3D reconstruction of MSCT and analyze the anatomical relationship between the injured part and the adjacent structure, which effectively overcomes the deficiencies of MRI and X-ray plain films. According to the MSCT findings of the study, vertebral fractures were shown as flattening of the vertebral body with a wedge-shaped appearance, and in 82 cases, the fracture line and displaced bone were visible, 4 of which with minor fractures showed no trabecular bone density on conventional MSCT, and after 3D reconstruction, morphological changes could be found, and thus, the diagnosis was confirmed. MSCT 3D reconstruction compensates for the deficit of MRI insensitivity to the cortical bone and clearly and intuitively reveals the fracture site. Scholars Saman et al. found that this modality also has good diagnostic value for determining the size and number of vertebral fracture fragments [24]. Based on the three-column concept, among the 100 patients included in this study, 52 cases had fracture at the anterior column of the spine, 28 cases had fracture at the middle column of the spine, and 20 cases had fracture at the posterior column of the spine; 24 cases had simple flexion compression fracture, 60 cases had burst fracture, 6 cases had seat belt fracture, and 10 cases had fracture dislocation. The accordance rate of combining plain film X-ray, MRI, and MSCT 3D reconstruction for fracture site was 100%, and that for fracture type was 98.0%, confirming that the combined examination can make their respective advantages complementary to each other and effectively improve the detection accuracy of spinal injuries.

In short, MRI can reveal bone marrow injury, ligament injury, soft tissue injury, and nerve root injury that cannot be visualized on X-ray plain films, and MSCT 3D reconstruction can clearly demonstrate the 3D relationship of spinal fracture displacement, fracture line course, and spinal injury. Plain film X-ray, as the basic method of diagnosing spinal injuries, still cannot be replaced nowadays, but MRI and MSCT can make up for the shortcomings of plain film X-ray and play a role in drawing on each other's strengths. For patients with negative X-ray results, MRI and MSCT can be used to observe the spinal injury comprehensively, which is conducive to reducing the disability rate and mortality rate of patients with spinal injuries.

## Figures and Tables

**Table 1:** Analysis of results of imaging examinations.

Group	MRI	MSCT	X-ray plain films	Joint examination
Anterior ligament injury	48	10	0	65
Posterior ligament injury	24	8	0	32
SCI	63	15	0	72
Soft tissue injury	76	86	20	86
Fracture line	92	95	78	95
Vertebral arch fracture	60	65	48	70
Nerve root injury	28	70	10	72

**Table 2:** Comparison of accordance rates of imaging examinations.

Group	MRI	MSCT	X-ray plain films	Joint examination
Fracture site	90 (90.0)	100 (100.0)	82 (82.0)	100 (100.0)
Fracture type				
Simple flexion compression fracture	20 (83.3)	22 (91.7)	18 (75.0)	24 (100.0)
Burst fracture	50 (83.3)	58 (96.7)	48 (80.0)	59 (98.3)
Seat belt fracture	4 (66.7)	5 (83.3)	3 (50.0)	5 (83.3)
Fracture dislocation	7 (70.0)	9 (90.0)	7 (70.0)	10 (100.0)

## Data Availability

The data supporting the findings of this study are available on reasonable request from the corresponding author.
